The article "RPE-derived exosomes rescue the photoreceptors during retina degeneration: an intraocular approach to deliver exosomes into the subretinal space" was published in 2021. Journal: Drug Deliv.

# RPE-derived exosomes rescue the photoreceptors during retina degeneration: an intraocular approach to deliver exosomes into the subretinal space

**DOI:** 10.1080/10717544.2020.1870584

**Published:** 2021-01-27

**Authors:** Yange Wang, Qian Zhang, Guoqing Yang, Yuanmeng Wei, Miao Li, Enming Du, Haijun Li, Zongming Song, Ye Tao

**Affiliations:** a Department of Ophthalmology, People’s Hospital of Zhengzhou University; Department of Physiology, Basic College of Medicine, Zhengzhou University, Zhengzhou, China; b Department of Clinical Aerospace Medicine, Fourth Military Medical University, Xi’an, China

**Keywords:** Subretinal delivery, neural degeneration, therapeutics

## Abstract

Retinal degeneration (RD) refers to a group of blinding retinopathies leading to the progressive photoreceptor demise and vision loss. Treatments against this debilitating disease are urgently needed. Intraocular delivery of exosomes represents an innovative therapeutic strategy against RD. In this study, we aimed to determine whether the subretinal delivery of RPE-derived exosomes (RPE-Exos) can prevent the photoreceptor death in RD. RD was induced in C57BL6 mice by MNU administration. These MNU administered mice received a single subretinal injection of RPE-Exos. Two weeks later, the RPE-Exos induced effects were evaluated via functional, morphological, and behavior examinations. Subretinal delivery of RPE-Exos efficiently ameliorates the visual function impairments, and alleviated the structural damages in the retina of MNU administered mice. Moreover, RPE-Exos exert beneficial effects on the electrical response of the inner retinal circuits. Treatment with RPE-Exos suppressed the expression levels of inflammatory factors, and mitigated the oxidative damage, indicating that subretinal delivery of RPE-Exos constructed a cytoprotective microenvironment in the retina of MNU administered mice. Our data suggest that RPE-Exos have therapeutic effects against the visual impairments and photoreceptor death. These findings will enrich our knowledge of RPE-Exos, and highlight the discovery of a promising medication for RD.

## Introduction

Retinal degeneration (RD) is a heterogeneous group of vision-threatening diseases that are characterized by progressive photoreceptors loss. The most common forms of RD are initiated by mutations in these genes closely related to photoreceptor function and metabolism (Chang et al., 2002; Scholl et al., 2016). The exact molecular pathways by which gene mutations lead to photoreceptor death have not been clearly characterized. Various studies employing a number of experimental models have shed light on substantial aspects in RD. It has been recognized that several pathological events include apoptosis, autophagy, and necrosis, occur during the process of RD (Boya et al., 2016). In particular, oxidative stress due to the exacerbating metabolism seems to be a significant influential factor in RD pathology. Up-regulation of oxidative markers and energetic dysfunction are early events involved in the photoreceptor death (Datta et al., 2017). Excessive oxidative stress produces bursts of reactive oxygen species (ROS), which will disturb the electron transport chain, cause damages to mitochondria, and eventually affects the survival of retinal neurons (Bellezza, 2018). Furthermore, the oxidative stress is associated with inflammatory response during retina degeneration. Oxidative stress can activate the retinal microglia and promote the release of inflammatory cytokines and chemokines in RD patients as well as animal models (Rashid et al., 2018). In this context, genetic and pharmacological strategies targeting the oxidative stress are designed to enhance photoreceptor survival in the degenerative retina. Researchers propose that antioxidants may elicit a better visual prognosis for RD patients (Limoli et al., 2020).

The article "RPE-derived exosomes rescue the photoreceptors during retina degeneration: an intraocular approach to deliver exosomes into the subretinal space" was published in 2021. Journal: Drug Deliv.

Retinal pigment epithelium (RPE) consists of a mono cell layer that separates blood vessels from neural retina and supports the survival light-sensitive photoreceptors. Due to its special anatomical location and function, the RPE accomplishes a pivotal role in maintaining retinal homoeostasis (Fuhrmann et al., 2014). RPE cells joint together via intercellular tight junctions, and block these free passages of ions and water. RPE also undertake a broad spectrum of physiological functions of the retina: scavenge of reactive oxidative species, nutrient delivery, ionic homeostasis, phagocytosis of cell debris, and production of nutritional cytokines. Impairments of RPE will cause excessive oxidative stress, mitochondrial destabilization, and activation of inflammatory response, all of which are implicated in the pathogenesis of RD (Ao et al., 2018). Mutations of RPE related genes would engender a series of conditions ranging from consecutive visual defects to severe phenotype of retinal dystrophies (Han et al., 2014).

RPE cells are readily sustainable in laboratory culture and suitable for cell transplantation (Nommiste et al., 2017). Recent advances in the surgical technique and transplantation instruments support the concept of RPE treatment as a regenerative strategy. Researchers have endeavored to assess the safety and effectiveness of RPE transplantation for RD patients or animal models (Alexander et al., 2015). They use a blunt needle or glass cannula to deliver either the RPE cell suspension, or a patch of RPE graft into the subretinal space. Although these attempts to transplant RPE into the appropriate anatomical space are largely successful, the outcomes are always far from satisfactory, because the transplantation techniques carry the risks of immunological rejection, surgical trauma, and cause disturbance of blood–retinal barrier (Cuevas et al., 2019). Previous studies have shown that implantation of RPE cells cause the multilayered fibrocellular scar, and the subsequent atrophy of photoreceptors overlying the implant (Kashani et al., 2018; Stanzel et al., 2019). Interestingly, RPE cells can secrete exosomes in a paracrine manner to influence neighboring cells (Locke et al., 2014). The role of exosomes in angiogenesis, apoptosis, autophagy, and inflammation has been well established. They have been delivered via intraocular, intranasal, intravenous, and other systemic routes to interfere with the pathological process of ocular diseases (Li et al., 2020).

The article "RPE-derived exosomes rescue the photoreceptors during retina degeneration: an intraocular approach to deliver exosomes into the subretinal space" was published in 2021. Journal: Drug Deliv.

RPE-derived exosomes (RPE-Exos) are extracellular vesicles which contain a set of genetic materials and proteins from their cells of origin (Biasutto et al., 2013). Due to their minuscule dimensions and lipid membrane, RPE-Exos can readily pass across retinal–blood barriers and deliver therapeutic factors into lesion. Compared with cell or graft transplantation, the subretinal delivery of RPE-Exo may cause less mechanical disruptions, and achieve better preserved retinal architecture. They hold promise for preventing photoreceptor loss and maintaining visual function due to their versatile biological activities, such as modulating immune responses, suppressing inflammatory responses, prompting cell differentiation, and inhibiting apoptotic cascades (Kannan et al., 2016; Li et al., 2020). When exposed to oxidative stress, RPE cells would secrete a higher quality of exosomes which are rich of phosphorylated signaling proteins. RPE cells also secrete αB-crystallin within exosomes upon stressed conditions, thereby maintaining favorable retinal environment and providing neuroprotection to neighboring cells (Sreekumar et al., 2010). On the basis of these findings, we intend to study the RPE-Exos induced effects on the RD models. We perform intraperitoneal injection in mice with a known apoptosis inducer, MNU, to build RD models. Subsequently, RPE-Exos was injected into the subretinal space of MNU administered mice. Our data show that the subretinal delivery of RPE-Exos can benefit photoreceptor survival and enhance the retinal responsiveness of RD models. These findings will enrich our knowledge of RPE-Exos, and highlight the discovery of an effective medication for RD.

## Materials and methods

### Exosomes isolation and characterization

ARPE-19 cells were plated in a T75 culture flask and cultured for 24 hours. When the cells reached 80% confluency, they were rinsed twice with phosphate-buffered saline (PBS) and incubated for 48 hours with freshly prepared complete medium. Then, the culture supernatants were collected, and the suspended cells were removed by centrifugation (300×*g*, 10 min, 4 °C). The culture supernatant was subjected to sequential centrifugation at 2000×*g* for 10 min, 10,000×*g* for 30 min, and 120,000×*g* for 70 min, and then filtered with a 0.22 μm filter (Guay et al., 2019; Jiang et al., 2020). Exosomes concentration was quantified by bicinchoninic acid protein Assay Kit (Biorega, Tianjin, China). The final concentration of exosomes derived from RPEs is 1.5 μg/μL. A transmission electron microscopy (TEM, JEM-1200EX, JEOL, Akishima, Japan) was used to examine the morphology of the exosomes. Potential surface markers were examined by western-blot analysis and flow cytometry assay. The extracted exosome preparations were stored at −80 °C and subjected to nanoparticle tracking analysis. A clean-disposable sample pool was chosen, and wiped with dust-free paper to ensure that no particle adhered to the outer tube wall in the light path. The exosomal solutions were slowly injected into the appropriately slant sample pool to avoid air bubbles. Then, the sample pool was put into the Nano series-Nano-ZS instrument to examine the size distribution and particle concentration of these particles.

The article "RPE-derived exosomes rescue the photoreceptors during retina degeneration: an intraocular approach to deliver exosomes into the subretinal space" was published in 2021. Journal: Drug Deliv.

### Animal modeling and drug delivery

Mice (C57/BL, age range 8–10 weeks, weighing between 21 and 25 g) were housed in the SPF animal facility (18–23 °C, 40–65% humidity). Each procedure involving animal handling was approved by Zhengzhou People’s Hospital and adhered to the ARVO statement for the Use of Animals in Ophthalmic and Vision Research. Four animal groups were included in this research: normal controls, MNU group, MNU + vehicle group, and MNU + RPE-Exos group. MNU (Sigma, St. Louis, MO; at the dose of 60 mg/kg) was injected intraperitoneally to induce RD in the mice. For treatment, the subretinal injection of RPE-Exos was performed instantly after MNU administration. One microliter PBS (vehicle) or 1 μL RPE-Exos were injected into the subretinal cavity. Procedures of subretinal injection followed a previous described method (Choi et al., 2018). Tobramycin ophthalmic ointment was applied to the conjunctival sac after surgery. The delivered therapeutic agents would produce bleb and partial retinal detachment (RD) between the neuroretina and RPE layer. The partial RD will reattach and become stable by two days post-injection (Qi et al., 2015). Two weeks after delivery, functional and morphological analysis was performed on these mice. In each examination section, eight animals were used for every animal group.

The article "RPE-derived exosomes rescue the photoreceptors during retina degeneration: an intraocular approach to deliver exosomes into the subretinal space" was published in 2021. Journal: Drug Deliv.

### Optokinetic behavior test

The visual responsiveness of mice was evaluated by their optomotor responses to moving sine wave gratings (Kretschmer et al., 2015). Briefly, stimulus gratings were projected on the wall of the machine under the control of a computer (OptoMotry CerebralMechanics, Lethbridge, Canada). Mice reflexively track the rotating virtual cylinders by moving their head if they could see the gratings clearly. The examiner could monitor the animal’s optomotor response via an infrared television camera located at the top of the testing box. The initial test parameters and protocols followed the instructions of the manufactures.

### Electroretinogram (ERG) examination

Mice were dark adapted overnight and were deeply anesthetized by an intraperitoneal injection of ketamine (80 mg/kg) and chlorpromazine (15 mg/kg, Shengda Animal Pharmaceutical, Jilin, China). Their pupils were dilated with tropicamide eye drops (Shenyang Xingqi, Shenyang, China). A platinum circellus electrode was placed in connect with the central cornea and a reference electrode was inserted beneath the cheek mucosa. Full-field light stimulus from the RETI port system (Roland Consult, Brandenburg, Germany) was used to induce the ERG responses. In this study, the scotopic responses were documented at the light intensity of 0.5 log cd-s/m^2^, while photopic recordings at the light intensity of 1.48 log cd-s/m^2^. The amplitude of a-wave was defined as the distance from baseline to a-wave trough, while the amplitude of b-wave was measured as the distance between trough and peak of each waveform.

### Spectral-domain optical coherence tomography (SD-OCT)

SD-OCT examination was performed on these anesthetized mice immediately after ERG examination. The mouse was moved onto on plate of Micron IV imaging system (Phoenix Research, Pleasanton, CA) after their pupils were dilated. Examiner adjusted the position of probe to produce horizontal volume scans until legible images appeared on the monitor screen. In each examination, three lateral scans were made starting 0.3 mm above the optic nerve head (ONH) meridian, at the ONH meridian and 0.3 mm below ONH meridian. A corresponding box was centered on the ONH, and the retinal thickness was measured at eight selected points within the scan (separated at the distance of 0.3 mm) using a software accessory kit. The obtained values were averaged for each mouse. The retina thickness of mouse eye was quantified by measuring the distance from the vitreal face of GCL to the apical face of the RPE.

The article "RPE-derived exosomes rescue the photoreceptors during retina degeneration: an intraocular approach to deliver exosomes into the subretinal space" was published in 2021. Journal: Drug Deliv.

### Multi electrode array (MEA) recording

The MED-64 system (Alpha MED Sciences, Osaka, Japan) was used to document the topographic electrical responses of mice (Xu et al., 2019). Briefly, retinal flat-mount patch was placed in to the center of the electrodes array of recording chamber. Light stimulus (with the mean intensity of 850 mcd-s/m^2^) was projected onto recording chip, there by triggering off the local field potentials (LFPs) of retinal neurons. Electrodes in the recording chip detected these electrical activities and then transmitted them into the computing monitor for further off-line analysis.

### Histological and immunohistochemical analysis

Eyeballs were collected from euthanized mice and were fixed in phosphate buffered paraformaldehyde (4%). These eyeballs were then dehydrated and optimum cutting temperature (OCT)-embedded. Hematoxylin–eosin staining was performed on the frozen sections. The nuclear layer (ONL) thickness was measured using the ImageJ software (Bethesda, MD). For immunohistochemistry, the retinal sections were blocked with 3% bovine serum albumin (BSA) at 37 °C for 30 min, and were incubated subsequently with primary antibodies (rabbit polyclonal cone opsin antibody 1: 400, Millipore, Billerica, MA) or peanut agglutinin (PNA) conjugated to a Alexa Fluor 488 (1: 200, Invitrogen, Carlsbad, CA) overnight at 4 °C. The retinal specimens were rinsed thoroughly, and then were incubated with Cy3-conjugated anti-rabbit IgG (1:400, Jackson ImmunoResearch Laboratories, West Grove, PA) and DAPI at 37 °C for 30 min. After washing with PBS, these retinal sections were observed using a Zeiss LSM 510 META microscope (Zeiss, Thornwood, NY) fitted with Axiovision Rel. version 4.6 software (Carl Zeiss AG, Oberkochen, Germany). All fluorescent images were captured using identical exposure settings to ensure consistent stable lighting throughout the image capture procedure. A background image of a blank slide was taken for each sample set and was subtracted from the corresponding sample image.

### Quantitative reverse transcription-polymerase chain reaction (qRT-PCR)

Total RNA was extracted from microglial cells mouse retinas using TRIzol reagent (Invitrogen, Carlsbad, CA) and reverse-transcribed to cDNA using a PrimeScript RT reagent kit (TaKaRa, Dalian, China). Reactions were performed with SYBR Green Master Mix on a real-time Touch PCR detection system (Tiangen Biotech, Reinach, Switzerland). The amplification program consisted of polymerase activation at 95 °C for 5 min and 50 cycles of denaturation at 95 °C for 1 min, annealing and extension at 59 °C for 30 seconds. Threshold cycle efficiency corrections were calculated, and melting curves were obtained using cDNA for each individual-gene PCR assay. The primers sets are listed in Table 1. The relative expression levels were normalized and quantified to obtain the ΔΔCT values for each sample.

The article "RPE-derived exosomes rescue the photoreceptors during retina degeneration: an intraocular approach to deliver exosomes into the subretinal space" was published in 2021. Journal: Drug Deliv.

**Table 1.** Primers sequences for mRNAs amplified in qRT-PCR.

Gene	Primer sequences
*Bax*	5′-AGCTCTGAACAGATCATGAAGACA-3′ (forward)
	5′-CTCCATGTTGTTGTCCAGTTCATC-3′ (reverse)
*Bcl-2*	5′-GGACAACATCGCTCTGTGGATGA-3′ (forward)
	5′-CAGAGACAGCCAGGAGAAATCAA-3′ (reverse)
*Caspase-3*	5′-ATG GGA GCA AGT CAG TGG AC-3′ (forward)
	5′-CGT ACC AGA GCG AGA TGA CA-3′ (reverse)
*TNF-α*	5′-CCC TCA CAC TCA GAT CAT CTT CT-3′ (forward)
	5′-GCT ACG ACG TGG GCT ACA G-3′ (reverse)
*IL-1β*	5′-AAACAGATGAAGTGCTCCTTCCAGG-3′ (forward)
	5′-TGGAGAACACCACTTGTTGCTCCA-3′ (reverse)
*IL-6*	5′-GCAAAGGGAAACTCACCA-3′ (forward)
*Calpain-2*	5′-AACACCTGTTTGGCTTTTAG-3′ (reverse)
	5′-CCCCAGTTCATTATTGGAGG-3′ (forward)
	5′-GCCAGGATTTCCTCATTCAA-3′ (reverse)

### Quantitative analysis of malondialdehyde concentration

A total bile acids colorimetric assay was used to measure the retinal malondialdehyde (MDA) concentration according to the guidance of the manufacturer’s protocol (Jiancheng Biotech Ltd., Nanjing, China). The MDA concentration was expressed as nmol/g retinal protein as described previously (Siu & To, 2002).

### Statistical analysis

Data are presented as mean and standard deviation. One-way ANOVA with Bonferroni’s post hoc analysis was used to analyze the differences among animal groups. A *p* value<.05 was considered statistically significant.

## Results

### RPEs-exosomes characterization

These particles derived from ARPE-19 cells were examined under electron microscopy (Figure 1(A)). These particles were put into the ZETASIZER Nano series-Nano-ZS instrument, and laser was projected on these samples. These particles could refract the scattering light. The extracted particles appeared as specific spheroidal shape with the diameters of approximately 40–100 nm (Figure 1(B)). Western blot assay was used identify the biomarkers of these particles (Figure 1(C)). We detected the expression of CD81 and TSG101, two biomarkers of exosomes, in these vesicles samples. Flow cytometry analysis showed that surface proteins CD63 and CD81 were expressed in these vesicles (Figure 1(D)). The positive rates of CD63 and CD81 are 69.9% and 74.9%, respectively. These findings suggest that these RPE-Exos were pure and could be used for subsequent therapeutic trials.

**Figure 1.** (A) Upper micrographs: particles derived from RPE appeared as specific spheroidal shape under electron microscopy. Bottom micrographs: the particles of scattering light were observed using the ZETASIZER Nano series-Nano-ZS instrument. When laser is projected on these samples, these white objects can refract the scattering light, indicating that the size of particles is uniform under dynamic light scattering. (B) Concentration and size distribution of the particles samples derived from RPEs by NTA. The diameters of extracted particles ranged between 40 and 100 nm. (C) Western blot assay was used to identify the biomarkers of these particles. The exosomes biomarkers CD81 and TSG101 were detected in these vesicles. (D) Flow cytometry analysis showed that surface proteins CD63 and CD81 were expressed in these vesicles (#1 and #2 represents two replicate samples derived from RPEs).

The article "RPE-derived exosomes rescue the photoreceptors during retina degeneration: an intraocular approach to deliver exosomes into the subretinal space" was published in 2021. Journal: Drug Deliv.

### Subretinal delivery of RPEs-exosomes retained retinal structure integrity

The MNU was used to induce RD in mice retinas. Histologically, by two weeks following MNU administration, the retinal architectures of the MNU group were severely disrupted without any nucleus in the ONL (Figure 2(A)). The retinal morphology of the MNU + vehicle group also underwent terrible destruction, since no improvement was found in these mice. Interestingly, the retinal cells of RPE-Exos treated group were organized in well-defined layers, which were similar to the architectures of the normal group. The mean ONL thickness of RPE-Exos treated group was significantly larger compared with MNU group (*p* < .01; *n* = 8). However, the mean ONL thickness of the vehicle treated group was not different from MNU group (*p* > .05; *n* = 8). OCT images collected from MNU group demonstrated the complete loss of ONL and the reduced thickness of total retinal layers (Figure 2(B)). OCT examination of the RPE-Exos treated group also revealed significant protective effects, seen as a thicker total retina thickness compared with MNU group (*p* < .01; *n* = 8). In general, subretinal delivery of RPE-Exos successfully alleviated the morphological injury in degenerative retina.

**Figure 2.** (A) RD was induced by an intraperitoneal injection of MNU. The subretinal injection of RPE-Exos was performed instantly after MNU administration. Morphological analysis was performed 2 weeks following treatment. Retinal architecture of MNU administered mice was effective preserved by RPE-Exos treatment. The mean ONL thickness of RPE-Exos treated group was significantly larger compared with MNU group. (B) OCT examination of the RPE-Exos treated group also revealed significant protective effects, seen as a thicker total retina thickness compared with MNU group (ANOVA analysis followed by Bonferroni’s post hoc analysis was performed, ^#^*p* < .01, for differences between groups; *n* = 8; GCL: ganglion cell layer; IPL: inner plexiform layer; OPL: outer plexiform layer; ONL: outer nuclear layer; INL: inner nuclear layer; OS: outer segments).

The article "RPE-derived exosomes rescue the photoreceptors during retina degeneration: an intraocular approach to deliver exosomes into the subretinal space" was published in 2021. Journal: Drug Deliv.

### Subretinal delivery of RPEs-exosomes rescued the visual function

ERG examination was performed to check the electrophysiology function of RPE-Exos treated mice. The representative ERG waveforms afforded a comparison of the waveforms (both scotopic and photopic phases) between the RPE-Exos and vehicle treated mice **(**Figure 3(A)). ERG data demonstrated better visual responsiveness in RPE-Exos treated mice, while no improvement was detected in these vehicle treated group. Quantified analysis showed that the b-wave amplitude was significantly larger in RPE-Exos treated group than that in the vehicle treated group (*p* < .01; *n* = 8; Figure 3(B)). The scotopic a-wave amplitudes were significantly larger in the MNU + RPE-Exos group than those in the MNU group (*p* < .01; *n* = 8). However, the scotopic a-wave amplitudes in the MNU + vehicle group were not significantly different from those in the MNU group (*p* > .05; *n* = 8). Consistent with the ERG data, optokinetic behavioral tests also showed that RPE-Exos induced therapeutic effects on the visual activity of MNU group. Both the visual acuity and contrast sensitivity in the RPE-Exos treated group were larger compared with the MNU group (*p* < .01; *n* = 8; Figure 3(C)). On the other hand, these parameters were not significantly different between the MNU + vehicle group and the MNU group (*p* > .05; *n* = 8). Collectively, these findings suggest that subretinal delivery of RPE-Exos rescued the visual function of RD models.

**Figure 3.** (A) Representative ERG waveforms demonstrated better visual responsiveness in RPE-Exos treated mice compared with MNU group. (B) The a- and b-wave amplitudes were significantly larger in RPE-Exos treated group than those in the vehicle treated group. (C) Optokinetic behavioral tests also showed that the visual acuity and contrast sensitivity in the RPE-Exos treated group were larger compared with the MNU group. (D) Immunohistochemistry work was performed on these retinal sections from central retina. Extensive punctate PNA staining was detected in the retinal sections of the RPE-Exos treated group. No PNA staining was found in the retinal sections of vehicle treated group. Abundant M- and S-cone opsin staining was also found in the retinal sections of RPE-Exos treated group (ANOVA analysis followed by Bonferroni’s post hoc analysis was performed, ^#^*p* < .01, for differences between groups; *n* = 8).

### Subretinal delivery of RPE-Exos rescued cone cells

Since the ERG data demonstrated critical improvement in the photopic vision RPE-Exos treated mice, we performed immunostaining experiments to examine the cone survival in these retinas (Figure 3(D)**)**. Extensive punctate PNA staining was detected in the retinal sections of the RPE-Exos treated group, indicating a substantial cone photoreceptors were preserved by RPE-Exos treatment. In the retinal sections of MNU group, no PNA staining was found since the outer and inner segments of the cone photoreceptors were severely disrupted. Furthermore, the viability of M- and S-cone subtypes was assessed using opsin antibodies. Abundant M- and S-cone opsin staining was found in the retinal sections of RPEs-Exos treated group. Conversely, these cone opsin staining disappeared in the vehicle treated group. These data indicated that the RPEs-Exos conferred extensive benefits on the M- and S-cone photoreceptors.

The article "RPE-derived exosomes rescue the photoreceptors during retina degeneration: an intraocular approach to deliver exosomes into the subretinal space" was published in 2021. Journal: Drug Deliv.

### Topographic quantification of the RPE-exosomes induced protective effects

MEA recording was performed to evaluate the electrical response of regional retina (Figure 4(A)). The mean LFPs amplitude of MNU group was significantly smaller compared with normal controls (*p* < .01; *n* = 8; Figure 4(B)). The mean LFPs amplitude of vehicle group was not significantly different from that of MNU group (*p* > .05; *n* = 8). Compared with MNU group, a significant improvement of LFPs amplitude was found in the RPE-Exos treated group (*p* < .01; *n* = 8). The recording field of MEA was set into three zones according to their distances to ONH: the central, the mid-peripheral, and the peripheral zone. Comparison analysis detected topographic differences among the three zones: LFPs amplitudes of central, the mid-peripheral, and peripheral zone in the RPEs-Exos treated mice were ∼18.3%, ∼42.4%, and ∼69.2% of the normal controls, respectively. Thus, the photoreceptors in peripheral region were more efficiently rescued by RPE-Exos treatment. Furthermore, the spontaneous firing frequency of MNU group increased significantly compared with normal controls (*p* < .01; *n* = 8; Figure 4(C)), suggesting that visual signal transmission was severely disturbed in these mice. On the other hand, the increase of spontaneous firing frequency was relatively slighter in the RPE-Exos treated group, suggesting that RPE-Exos treatment could enhance the efficiency of visual signal transmission.

**Figure 4.** (A) As shown in the MEA recording, the electrical response of retina was affected remarkably by MNU toxicity. However, the LFPs of the MNU + RPE-Exos group were effectively preserved. (B) Comparison analysis showed that the LFPs amplitude was significantly larger in the MNU + RPE-Exos group than that in the MNU group. In particular, these photoreceptors in peripheral region were more efficiently rescued by RPE-Exos treatment. (C) MNU administration also affected the firing activities of retinal neurons, as evidenced by an elevated firing frequency in the MNU group. Conversely, the increase of spontaneous firing frequency was relatively slighter in the MNU + RPE-Exos group (ANOVA analysis followed by Bonferroni’s post hoc analysis was performed, ^#^*p* < .01, for differences between groups; *n* = 8).

The article "RPE-derived exosomes rescue the photoreceptors during retina degeneration: an intraocular approach to deliver exosomes into the subretinal space" was published in 2021. Journal: Drug Deliv.

### RPE-exosomes ameliorated the inflammatory and apoptotic response

The relative mRNA levels of apoptotic factor and pro-inflammatory cytokine in retina were investigated by RT-PCR. In comparison with normal controls, the mRNA levels of pro-inflammatory cytokines, including IL-1β, IL-6, TNF-α, and MCP-1 increased significantly higher in the MNU group (*p* < .01; *n* = 8; Figure 5), indicating that inflammation was involved in the pathogenesis of retina degeneration. On the other hand, the mRNA levels of these pro-inflammatory cytokines reduced significantly in the RPE-Exos treated group than those the MNU group (*p* < .01; *n* = 8). The mRNA levels of Bax, Calpain-2, and Caspase-3 decreased significantly in RPE-Exos treated group than those in the MNU group (*p* < .01; *n* = 8), whereas the mRNA level of bcl-2 increased significantly (*p* < .01; *n* = 8). Endoplasmic reticulum stress and the subsequent Ca^2+^ overload can activate the calcium dependent cysteine proteases known as Calpain-2 (Cuenca et al., 2014). Calpains-2 can work collaboratively with other mediators to amplify the apoptotic signal. Activation of Calpains-2 is considered an important caspase-independent apoptotic pathway in the photoreceptor degeneration of RD (Kanan et al., 2007; Zhang et al., 2017). Our data suggest that RPE-Exos may rescue the photoreceptors by inhibiting the caspase-independent apoptotic pathway. MDA is a stable metabolite of lipid peroxidation, and the retinal level of MDA has been examined to quantify the oxidative response (Ola et al., 2019). Analysis of retinal MDA concentration demonstrated a significant reduction in the RPE-Exo treated group than that in the MNU group (*p* < .01; *n* = 8). These data suggested that RPE-Exos therapy mitigated the oxidative stress of degenerative retinas.

**Figure 5.** (A) The mRNA levels of these pro-inflammatory cytokines, including IL-1β, IL-6, TNF-α, MCP-1, reduced significantly in the RPE-Exos treated group than those the MNU group. The mRNA levels of Bax, Caspase-3, and Calpain-2 decreased significantly in MNU + RPE-Exos group than those in the MNU group, whereas the mRNA level of bcl-2 increased significantly. Analysis of retinal MDA concentration demonstrated a significant reduction in the RPE-Exo treated group than that in the MNU group, indicating that RPE-Exos can alleviate the oxidative stress in retina (ANOVA analysis followed by Bonferroni’s post hoc analysis was performed, ^#^*p*<.01, for differences between groups; *n* = 8).

The article "RPE-derived exosomes rescue the photoreceptors during retina degeneration: an intraocular approach to deliver exosomes into the subretinal space" was published in 2021. Journal: Drug Deliv.

## Discussion

RPE cells support the photoreceptors by releasing nano-sized exosomes into the intercellular matrix under physiological and pathological conditions. These RPE-Exos act as vital mediators during intercellular communication by delivering membrane proteins, mRNAs, and miRNAs to recipient cells (Biasutto et al., 2013; Klingeborn et al., 2018). This study investigates the RPE-Exos induced therapeutic effect on an experimental RD model. We delivered RPE-Exos into the subretinal space of MNU administered mice, and found that RPE-Exos treatment alleviates the photoreceptor apoptosis, suppresses the expression levels of inflammatory cytokine, and enhances the visual responsiveness. The heterogeneity of RD is challenging for any therapy. On the other hand, each animal model has its limitation and cannot perfectly mimic the pathological process in human patients. In this study, only one type of murine RD model was used to test the efficacy of RPE-exosomes. This should be recognized as a drawback of this study. In order to prevent the over-exaggeration of the RPE-exosomes induced beneficial effects, more studies are needed to evaluate the efficiency, safety, and technical challenges appropriately. The therapeutic effects of RPE-Exos in this study are achieved through subretinal injection, implying that intraocular delivery approach may help them reach the site of lesion. Typically, exosome membrane is consolidated enough to protect their functional cargos from external disturbances (Skotland et al., 2019). Through this way, functional materials are transported from RPE to host cells, leading to the production of proteins with versatile biological functions. The MNU administered mouse is a chemically induced RD model with rapidly progressive dynamics. Typically, this animal model entirely lost ERG amplitudes and photoreceptors one week after MNU administration (Tsubura et al., 2010). The modeling mechanism should be ascribed to the principal DNA alkylation that is induced by the MNU toxicity. MNU can produce 7MeG and 3MeA DNA lesions, both of which are alkyladenine DNA glycosylase (Aag) substrates (Tsubura et al., 2011). The base excision repair machinery cannot work efficiently enough when the Aag loses its ability to function, and the photoreceptor would die due to these DNA alterations. As the DNA damage acts as a critical mechanism underlying the MNU induced photoreceptor death, it is tempting to speculate that RPE-Exos may repair the DNA damages of photoreceptor. Future investigation is warranted to decide whether the RPE-Exos affects the DNA alkylation.

The article "RPE-derived exosomes rescue the photoreceptors during retina degeneration: an intraocular approach to deliver exosomes into the subretinal space" was published in 2021. Journal: Drug Deliv.

Progressive photoreceptor loss is the hallmark of RD patients with different genetic backgrounds (Risenhofer et al., 2017). Although the causative genetic mutations are often known, the underlying mechanisms leading to photoreceptor death remain poorly defined. Accumulating evidences show that apoptosis is a common feature of RD pathogenesis (Doonan & Cotter, 2004). The intraocular delivery of pharmacological agent or gene vector represents a promising therapeutic strategy against RD (Fischer, 2016; Mead & Tomarev, 2017; He et al., 2018). As evidenced by animal and clinical trials, these therapeutic molecules could retard the photoreceptor apoptosis, and ameliorate the vision loss once they are delivered efficiently into the eye (CATT Research Group et al., 2011; Athanasiou et al., 2018). However, the enormous heterogeneity implied in RD pathogenesis is challenging for any therapeutic approach. In this study, we show that the subretinal delivery of RPE-Exos mitigates the mRNA levels of apoptotic factors. It has been speculated that RPE-Exos may contain components influencing the caspase-mediated apoptotic cascades. Thus inhibiting the photoreceptor apoptosis by RPE-Exos might be developed into a promising therapy for RD. Retina is characterized by the active metabolic rate, and intense oxygen consumption. Treatment with antioxidants alleviates the RD progression in patients and animal models. Herein, we show that subretinal delivery of RPE-Exos reduces the level of oxidative marker in retinas. It is conceivable that RPE-Exos would provide a beneficial environment for retinal neurons. When the photoreceptors are exposed to excessive oxidative stress, RPE-Exos can internalize to mitochondria, endoplasmic reticulum, and nucleus to initiate anti-oxidative events (Locke et al., 2014). Previous studies have shown that RPE-Exos contain a myriad of αB-crystallin, a mitochondrial and cytosolic protein with potent anti-oxidative capacity (Kannan et al., 2016). Accordingly, RPE-Exos might act as vectors in RD therapy through its potency of shuttling antioxidants. Inflammation is also correlated with the photoreceptor death in RD pathogenesis (Kauppinen et al., 2016). In this study, we show that MNU toxicity can enhance the mRNA levels of pro-inflammatory cytokines, such as TNF-α, IL-1β, and MCP-1. The over-expression of inflammatory cytokines is also detected in the vitreous fluid of RD patients (McMurtrey & Tso, 2018; Massengill et al., 2018). These findings highlight the possibility that inflammatory response happens to debilitate the photoreceptors regardless of the etiological cause during RD process. It is noteworthy that modulating inflammatory response would alleviate the functional and morphological damages in RD (Rashid et al., 2018). Exosomes represent an emerging therapeutic agent that provided new insights into the manipulation of inflammatory response. They act as immune response mediators with specific roles in antigen presentation (Théry et al., 2009). Moreover, the distinctive properties of exosomes make them appropriate carriers for the delivery of anti-inflammatory biomolecules (Srivastava et al., 2016). Researchers propose that exosomes may be developed into therapeutic modalities against these inflammation related diseases. TNF-α acts as an upstream mediator for photoreceptor death, since it can trigger off inflammatory response by recruiting CD11b-positive phagocytes and induce apoptosis by activating caspase-8 (Nakazawa et al., 2011). On the contrary, inhibition of TNF-αexpression would up-regulate the autophagy level and facilitate photoreceptor survival (Xie et al., 2017). MCP-1 is cytotoxic to photoreceptor cells since it can recruit and activate the macrophages and microglia (Nakazawa et al., 2007). IL-1β is another mediator of inflammatory response which exerts neurotoxic effects on photoreceptors (Yoneda et al., 2001). The exact mechanism by which RPE-Exos exert these beneficial effects remains to be elucidated. Retinal glia cells such as microglia, astrocytes, and Müller cells, can provide essential metabolic and structural support to photoreceptors, and control the composition of the surrounding microenvironment (Massengill et al., 2018). Once these glia cells are activated by external stimulus, they would fulfill macrophage function, and release inflammatory factors. These factors would exacerbate neuroinflammation and hasten retinal neuron death (Cuenca et al., 2014). An increase in pro-inflammatory cytokine levels is a hallmark of various RD animal models (Zeng et al., 2005; Rashid et al., 2019). Therefore, inflammatory response is secondary to initial injury following the MNU administration. Under acute conditions, an inflammatory response triggered by retinal microglia promotes neuroprotection, and only prolonged exposure leads to excessive amounts of proinflammatory factors that in turn cause exacerbated tissue injury (Rashid et al., 2019). Accordingly, RPE-Exos may not even have a direct anti-inflammatory effect, simply because fewer cells in the treated retinas have undergone degenerative processes. Further studies are necessary to decide whether the RPE-Exos can inhibit the inflammatory response.

The article "RPE-derived exosomes rescue the photoreceptors during retina degeneration: an intraocular approach to deliver exosomes into the subretinal space" was published in 2021. Journal: Drug Deliv.

Cone photoreceptor is charge of visual acuity and color vision of mammal. The impaired color/contrast sensitivity due to the progressive of cone photoreceptors is a critical event in RD pathology (Liutkevičienė et al., 2014). Mouse retina has two cone populations that can be distinguished by the special visible light spectrum to which they are sensitive (Allen et al., 2011; Cunea et al., 2014). The S-cones are sensitive to the short wavelength (blue) light stimulus, while the M cones are sensitive to the medium wavelengths (red) light stimulus. Typically, the well characterized antibodies can bind to the opsin protein in outer segments, thereby distinguishing the two cone populations (Narayan et al., 2019). We show that both the M- and S-cone photoreceptors are rescued by RPE-Exos. These findings are consistent with immunostaining assays employed the PNA which specifically labels cone matrix sheaths. The RPE-Exos not only induce beneficial effects on cone viability, but also yield functional benefits as corroborated in the photopic ERG examinations. Previous studies suggest a close relationship between rod viability and cone survival in degenerative retinas (Narayan et al., 2016; Sahel & Léveillard, 2018). An increment in the rate of rod viability would promote a substantially longer survival of cone. It is possible that the RPE-Exos mediated beneficial effects on rod photoreceptors would propagate subsequently to cone photoreceptors. In rodent retinas, cone photoreceptors distribute primarily as a ring in the equatorial retina, which is different from the fovea dependence on cones in human (Szél et al., 1996). Thus, the RPE-Exos induced beneficial effects on cones should be further validated by clinical trials.

MEA is a valuable tool to evaluate the effects of therapeutic agents on different locations of retina (Soto et al., 2020). The delicate electrodes of MEA are highly sensitive to the electrical activities of retinal neurons. In this study, we show that RPE-Exos treatment induces regional preservation on the retina of MNU administered mice. Typically, the MNU induced photoreceptor degeneration is not homogeneous: the damage in the central region is relatively more severe than that in the peripheral region (Boudard et al., 2010). Since the photoreceptors in the central retina are more sensitive to the MNU toxicity, it is well accepted that the photoreceptors in the peripheral regional would be more readily rescued by therapeutic agents (Chen et al., 2016). These topographic causes should be responsible for the differential regional preservation by RPE-Exos.

In conclusion, we show that subretinal delivery of RPE-Exos can ameliorate the photoreceptor loss and enhance the visual responsiveness of MNU administered mice. RPE-Exos confer these beneficial effects by suppressing apoptosis and relieving the oxidative damage. RPE-Exos act as critical regulator of photoreceptor apoptosis and provided a potential therapeutic agent for retinal disorders like RD. Further investigations are necessary to determine the safety and efficiency of RPE-Exos treatment, and to elucidate the specific cytokines with their working mechanisms.
